# Comparison of Diagnostic Performance between Perfusion-Related Intravoxel Incoherent Motion DWI and Dynamic Contrast-Enhanced MRI in Rectal Cancer

**DOI:** 10.1155/2021/5095940

**Published:** 2021-07-29

**Authors:** Ming Li, Xiaodan Xu, Kaijian Xia, Heng Jiang, Jianlong Jiang, Jinbing Sun, Zhihua Lu

**Affiliations:** ^1^Department of General Surgery, Changshu Hospital Affiliated to Soochow University, Changshu No.1 People's Hospital, Changshu, 215500 Jiangsu Province, China; ^2^Department of Gastroenterology, Changshu Hospital Affiliated to Soochow University, Changshu No.1 People's Hospital, Changshu, 215500 Jiangsu Province, China; ^3^Department of Central Laboratory, Changshu Hospital Affiliated to Soochow University, Changshu No.1 People's Hospital, Changshu, 215500 Jiangsu Province, China; ^4^Department of Radiology, Changshu Hospital Affiliated to Soochow University, Changshu No.1 People's Hospital, Changshu, 215500 Jiangsu Province, China

## Abstract

This study was aimed to determine the diagnostic performance of perfusion-related parameters derived from intravoxel incoherent motion diffusion-weighted imaging (IVIM-DWI) by comparing them with quantitative parameters from dynamic contrast-enhanced magnetic resonance imaging (DCE-MRI) based on differentiation grades of rectal cancer. We retrospectively analyzed 98 patients with rectal cancer. Perfusion-related IVIM parameters (*D*^∗^, *f*, and *f*·*D*^∗^) and quantitative DCE parameters (*K*^trans^, *K*_ep_, *V*_*e*_, and *V*_*p*_) were obtained by plotting the volume-of-interest on in-house software. Furthermore, we compared the difference and diagnostic performance of all well-moderately and poorly differentiated rectal cancer parameters. Finally, we analyzed the correlation between those DCE and IVIM parameters and pathological differentiation grade. The values of *f*, *K*^trans^, and *K*_ep_ significantly differentiated poor and well-moderate rectal cancers. *K*^trans^ achieved the highest area under the curve (AUC) value compared to perfusion-related IVIM and DCE parameters. Furthermore, *K*^trans^ showed a better correlation with pathological differentiation grade than *f*. The diagnostic efficiency of DCE-MRI was greater than perfusion-related IVIM parameters. The *f* value derived from perfusion-related IVIM offered a diagnostic performance similar to DCE-MRI for patients with renal insufficiency.

## 1. Introduction

Dynamic contrast-enhanced magnetic resonance imaging (DCE-MRI) is a quantitative technique that measures the capillary blood perfusion parameters of the tissue using intravenous contrast media and evaluates tissue properties such as capillary permeability and extracellular volume fraction that indirectly reflect the microcirculation and hemodynamics in the tissue [1]. Previous studies have demonstrated the efficiency of DCE-MRI in preoperative diagnosis of rectal cancer [2, 3], determining malignant inner wall irregularity in cystic-cavitary lung lesions [4] and evaluating disease activity of juvenile idiopathic arthritis [5]. However, DCE-MRI is not suitable for patients with contraindication to contrast media.

Intravoxel incoherent motion diffusion-weighted imaging (IVIM-DWI) collects multiple images containing low *b* values without using intravenous contrast media and analyzes them using a biexponential model. Quantitative parameters derived from IVIM-DWI can separate true molecular diffusion from the motion of water molecules [6], including pure diffusion coefficient (*D*), which represents the true tissue cellularity and diffusion; pseudo diffusion coefficient (*D*^∗^), which represents incoherent microcirculation; and perfusion fraction (*f*), which represents the number of protons linked to microcirculation [7]. *D*^∗^ and *f* are parameters related to perfusion. The clinical utility of IVIM-DWI has been established in a variety of tumors [7–10]. *D* values derived from IVIM-DWI demonstrated superior performance compared with ADC value, and perfusion-related IVIM parameters showed a correlation with quantitative parameters from DCE-MRI. Therefore, IVIM-DWI is suitable for patients with renal impairment. However, further research is still needed to compare the diagnostic performance of perfusion-related IVIM parameters and quantitative parameters from DCE-MRI.

Therefore, this study compared the diagnostic performance of perfusion-related parameters derived from IVIM-DWI with quantitative parameters derived from DCE-MRI based on differentiation grades of rectal cancer.

## 2. Materials and Methods

### 2.1. Patients

Our institutional review board approved this retrospective study and waived the requirement to obtain written informed consent. Selection criteria were as follows: (1) MRI examination including high-resolution T2WI, multiple *b* value DWI, and DCE-MRI and (2) the availability of pathology reports of surgical specimens. A total of 128 consecutive patients were enrolled between October 2016 and February 2021. Among these patients, 30 patients were excluded because of (1) poor image quality on T2WI, multiple *b* value DWI, and DCE-MRI (*n* = 19), (2) preoperative chemoradiotherapy (*n* = 6), and (3) other especial pathological conditions, such as mucinous adenocarcinoma (*n* = 5). Finally, 98 patients were included in the study.

### 2.2. MRI Technique

All patients were scanned with a 3.0-T MRI system (Intera Achieva 3.0 T TX, Philips Medical System, Best, the Netherlands) with a 16-channel phased-array surface coil. The patients underwent enema before MR imaging to reduce gas-induced artifacts in the rectum. Each patient received 10 mg anisodamine (Hangzhou Minsheng Pharmaceuticals Co. Ltd., Zhejiang, China) intramuscularly 10 minutes prior to the scan to minimize bowel peristalsis. The MRI protocol included the following parameters: (1) axial T1-weighted turbo spin-echo (TSE) (TR/TE = 550/10 ms, slice thickness = 6 mm, slice gap = 1.5 mm, field of view (FOV) = 300 × 300 mm, matrix = 376 × 336, number of excitations (NEX) = 2) (2) axial T2-weighted (T2W) fat suppression TSE (TR/TE = 3554/80 ms, slice thickness = 6 mm, slice gap = 1.8 mm, FOV = 300 × 379 mm, matrix = 376 × 374, NEX = 1), (3) high-resolution sagittal T2W TSE (TR/TE = 3577/70 ms, slice thickness = 3 mm, slice gap = 0 mm, FOV = 240 × 240 mm, matrix = 300 × 266, NEX = 3), (4) high-resolution oblique coronal T2W (TR/TE = 3000/75 ms, slice thickness = 2 mm, slice gap = 0 mm, FOV = 180 × 180 mm, matrix = 300 × 218, NEX = 3), and (5) high-resolution oblique axial T2W (TR/TE = 3000/75 ms, slice thickness = 3 mm, slice gap = 0 mm, FOV = 180 × 180 mm, matrix = 368 × 273, NEX = 3). The oblique coronal T2WI was parallel to the tumor axis. Moreover, as identified on sagittal T2WI, the oblique axial T2WI was perpendicular to the tumor axis.

We performed multiple *b* value DWI in a single-shot spin-echo echo-planar-imaging sequence in the orientation similar to axial oblique T2WI with the following parameters: TR/TE = 2750/76 ms, slice thickness = 3 mm, slice gap = 0 mm, FOV = 220 × 220 mm, matrix = 112 × 108, NEX = 2, and nine *b* values (0, 10, 20, 50, 100, 200, 500, 800, and 1000 s/mm^2^).

The DCE T1W THRIVE sequence was performed with the same orientation as axial oblique T2WI with the following parameters: TR/TE = 6.9/3.5 ms, slice thickness = 3 mm, slice gap = 0 mm, FOV = 220 × 220 mm, matrix = 184 × 182, NEX = 1, flip angle 10°, number of slices 64, and temporal resolution 5.3 seconds. The baseline T1 map was calculated using three precontrast T1-weighted fast field echo sequences with different flip angles (5°, 10°, and 15°, respectively) as references. These three precontrast reference series were similar to the DCE sequences. Each patient received a gadodiamide injection (Omniscan; Ge Healthcare, Ireland) intravenously at a flow rate of 2.5 ml/s (a dose of 0.2 ml/kg of body weight) during the scan.

### 2.3. Image Analysis

A focal mass or irregular wall thickening with intermediate-signal intensity on T2WI, hyperintensity on DWI with *b* value of 1000 s/mm^2^, and corresponding hypointensity on grey-scale ADC map were the criteria for rectal cancer. Two experts (Ming Li and Heng Jiang) manually drew the regions of interest (ROIs) slice by slice to cover as much of the entire tumor area as possible while excluding necrosis, cysts, and gas areas and keeping the ROIs on DWI and DCE consistent. When both of these experts disagreed, the third expert (Zhihua Lu) made the decision. An example of the placement of ROIs is shown in Figure 1.

IVIM-DWI raw data were postprocessed using an image analysis software FireVoxel that is based on Le Bihan's biexponential model [11]:

(1) $$\begin{array}{c} S_{b}/S_{0}=\left(1-f\right)\exp\left(-bD\right)+f\exp\left(-bD*\right), \end{array}$$

where *S*_*b*_ is the signal intensity in the pixel with diffusion gradient *b* value, *S*_0_ is the signal intensity in the pixel with *b* value of 0 s/mm^2^, *D* is the true diffusion representing pure molecular diffusion, *f* is the fractional perfusion representing microcirculation, and *D*^∗^ is the pseudodiffusion coefficient. The MATLAB software was used to calculate the average *D*^∗^ and *f* values in each pixel.

We analyzed DCE-MRI using the pharmacokinetic Extended Tofts Linear model. Furthermore, using the Omni Kinetics software (GE Healthcare, Shanghai, China), we quantitatively analyzed DCE. After importing the dynamic enhancement sequence, three precontrast T1-fast field echo sequences with different flip angles were imported. We drew the internal iliac artery vessel to obtain the time–concentration curve of the blood supply vessel as the arterial input function and used this curve as a reference. Moreover, the pseudocolor images of *K*^trans^, *K*_ep_, *V*_*e*_, and *V*_*p*_ and the average value of each parameter were analyzed.

### 2.4. Statistical Analysis

We analyzed our data statistically using the SPSS and MedCalc software. We estimated the distribution of all quantitative parameters using the Kolmogorov–Smirnov test. Normally distributed data were presented as mean ± standard deviation, whereas abnormally distributed data were presented as median value and interquartile range. To compare well-moderately differentiated and poorly differentiated tumors on all quantitative parameters, we used the independent sample *t*-test or Mann–Whitney *U*-test. Furthermore, we analyzed the diagnostic performance for well-moderately differentiated and poorly differentiated tumors using the receiver operating characteristic (ROC) curve. The correlations between those DCE and IVIM parameters and pathological differentiation grade, as well as between perfusion-related parameters of IVIM and DCE parameters, were evaluated using Spearman correlation analysis. We calculated the intraclass correlation coefficients (ICC) to determine the interobserver agreement between the measurement values of two experts. The ICC value of 0.00–0.20 demonstrated a poor agreement, 0.21–0.40 fair agreement, 0.41–0.60 moderate agreement, 0.61–0.80 good agreement, and 0.81–1.00 excellent agreement.

## 3. Results

### 3.1. Clinical and Pathological Findings

This study enrolled 98 patients, of which 60 were male and 38 female. The median age of patients was 66 years (range, 41–89 years). According to the histopathological analysis, 8 tumors were pT1, 32 tumors were pT2, 50 tumors were pT3, and 8 tumors were pT4. 56 patients were staged as N0, 26 patients were staged as N1, and the remaining 16 patients as N2. The differentiation grades of rectal cancer according to pathological results were as follows: well-differentiated in 6 patients, moderately differentiated in 51 patients, and poorly differentiated in 41 patients. Patients were divided into two groups. The first group included 57 patients with well-moderately differentiated grades, and the second group 41 patients with poorly differentiated grades.

### 3.2. Correlations between Perfusion-Related IVIM and DCE Parameters

There was a weak correlation between *f* and *K*_ep_ (*r* = 0.279, *p* = 0.005). However, no correlation was found among other perfusion-related IVIM and DCE parameters.

### 3.3. Perfusion-Related IVIM and DCE Parameters

Table 1 summarizes the comparison between well-moderately differentiated and poorly differentiated tumors using perfusion-related IVIM and DCE parameters. *f*, *K*^trans^, and *K*_ep_ were significantly higher in the group with poor differentiation than in the group with well-moderate differentiation (*p* < 0.001, *p* < 0.001, *p* = 0.002, respectively). There were no significant differences in *D*^∗^, *f*·*D*^∗^, *V*_*e*_, and *V*_*p*_ between the two groups.

### 3.4. Comparison of Diagnostic Performance of Perfusion-Related IVIM and DCE Parameters

The diagnostic efficiency of statistically significant perfusion-related IVIM and DCE parameters to discriminate poorly differentiated tumors is presented in Table 2. Among DCE parameters, *K*^trans^ had a higher AUC (77.5%) with a sensitivity of 85.4% and a specificity of 63.2% (Figure 2), whereas *K*_ep_ had a lower AUC of 71% with sensitivity and specificity of 92.7% and 49.1%, respectively. Among perfusion-related IVIM parameters, *f* had an AUC of 72.8% with a sensitivity of 92.7% and a specificity of 43.9%. Furthermore, *K*^trans^ derived from DCE parameters had a greater correlation with pathological differentiation grade (*r*_*s*_ = 0.471) than *f* derived from perfusion-related IVIM parameters (Table 3).

### 3.5. Interobserver Agreement

The assessment of interobserver agreement between the two radiologists by ICC revealed excellent agreements for all parameters derived from perfusion-related IVIM and DCE (Table 1).

## 4. Discussion

This study found that parameters *f*, *K*^trans^, and *K*_ep_ significantly distinguished poorly and well-moderately differentiated rectal cancer. *K*^trans^ had the highest AUC value compared with other perfusion-related IVIM and DCE parameters. Furthermore, *K*^trans^ showed a better correlation with pathological differentiation grade than *f*.

Although the imaging principles of IVIM-MRI and DCE-MRI vary, the basic theories are based on capillary permeability and hemodynamics hypotheses. Therefore, the relationship between perfusion-related IVIM and quantitative DCE-MRI parameters has been a topic of interest for researchers. Previous studies [12–15] have found that the perfusion-related IVIM parameters have a moderate to strong correlation with quantitative DCE-MRI parameters, suggesting that they can be used to diagnose and assess various tumors. In our study, we found a weak correlation between *f* and *K*_ep_ parameters. However, there was no correlation between *D*^∗^or *f*·*D*^∗^ and any quantitative DCE-MRI parameters, which may be attributed to several reasons. First, other factors such as microvessel anatomy, blood vessel permeability [16], and microvessel density [17] also affect the *f* value. Second, *K*^trans^ is affected by both blood volume and microvascular permeability. Third, the *D*^∗^ value may represent more than one physiological process, such as gland secretion and fluid flow in capillaries [18].

The *D*^∗^ value of perfusion-related IVIM parameters indicates a perfused capillary microcirculation in the tissue. The *f* value is related to the capillary blood volume and represents the rate of diffusion related to microcirculation perfusion in the respective voxel of interest compared to total diffusion. Moreover, *f*·*D*^∗^ allowed the estimation of relative perfusion or blood flow in the tumor microcirculation, which was previously thought to depend on the interaction among the microvascular anatomy, vascular permeability, and blood flow dynamics [19]. Our results showed that the *f* value in the poorly differentiated tumors was significantly higher than the well-moderately differentiated tumors. This may be because the permeability of immature blood vessels and capillaries increased with the increased malignancy of the tumor. This is in line with the results of another study [20], which found a significant correlation between *f* value and blood vessel count and microvessel density. However, Sun et al. [20] and Lu et al. [21] found that the *f* value gradually decreased with the increasing degree of malignancy. The differences in results between this study and others may be related to the increase in the complexity of the microvessels in the tumor as the degree of malignant increases.

The DCE-MRI quantitative parameters objectively assess the characteristics of microcirculation perfusion and microvessels in tissues. *K*^trans^ represents the rate of contrast media transporting through the vascular endothelium to the extravascular extracellular space (EES). *K*_ep_ is the opposite of *K*^trans^, and *K*^trans^ and *K*_ep_ represent the amount of microvascular perfusion in the tissue as well as the penetrated area of the blood vessel. Our findings revealed that *K*^trans^ and *K*_ep_ were significantly higher in rectal cancer with poor differentiation than that with well-moderate differentiation. This is because the structure and function of tumor neovascularization become impaired with the increase in the degree of malignancy of the tumor, resulting in higher permeability and blood flow in tumors with higher malignancy. This result is consistent with the findings of another study [2]. *V*_*e*_ is the size of EES, which reflects the percentage of contrast media concentration in the entire voxel in EES. The mixing of blood volume and plasma flow is represented by *V*_*p*_. In our study, the *V*_*e*_ and *V*_*p*_ values showed no significant difference between poor differentiation and well-moderate differentiation. This can be attributed to scan time and the tumor–node–metastasis (TNM) stage.

The ROC curves analysis revealed that *K*^trans^ achieved the highest AUC value for distinguishing between tumors with poor differentiation and those with well-moderate differentiation. Furthermore, Spearman correlation analysis showed that *K*^trans^ had a better correlation with pathological differentiation grade than *f*.

Before considering the implications of the findings of this study, it is important to consider some of the limitations. First, the sample size of well-differentiation tumors is small and insufficient. Patients with moderately differentiated grades will have a different prognosis. The sample size must be large, and the group must be refined to obtain better and significant results. Second, the selection of *b* value affects IVIM-MRI parameters. At present, there is no standard reference for the value and number of *b* values. Further research is needed to optimize the *b* value. Third, our study did not analyze the correlation between perfusion-related IVIM and DCE-MRI parameters and immunohistochemical findings (microvessel density and vascular endothelial growth factor). We will conduct a more in-depth analysis of comparison in the follow-up study.

## 5. Conclusion

In conclusion, our study showed that DCE-MRI had greater diagnostic accuracy than perfusion-related IVIM parameters. Especially, the *K*^trans^ derived from DCE-MRI parameters was the optimal parameter for diagnostic efficiency. Moreover, the *f* value derived from perfusion-related IVIM offers similar diagnostic performance to DCE-MRI for patients with renal insufficiency.

## Figures and Tables

**Figure 1:** A 48-year-old woman with rectal adenocarcinoma was performed by IVIM and DCE. (a) High-resolution oblique axial T2W showed intermediate-signal intensity lesion (white arrow). (b) DWI (b = 1000 s/mm^2^) showed a hyperintensity lesion (white arrow). (c) ADC map showed a hypointensity lesion (white arrow). (d) DCE-MRI showed an abnormal enhanced lesion (white arrow). (e) ROI was manually drawn to cover as much of the entire tumor area as possible (white circle).

**Figure 2:** ROC curves are shown the diagnostic performance of perfusion-related IVIM and DCE parameters for discriminate poor differentiation tumor.

**Table 1:** Comparison of perfusion-related IVIM and DCE parameters between well-moderate differentiation and poor differentiation tumor.

Parameters	Well-moderate differentiation (*n* = 57)	Poor differentiation (*n* = 41)	*P* value	ICC
*D* ^∗^(×10^−3^ mm^2^/s)	87.15 ± 14.46	82.95 ± 19.71	0.252	0.824
*f* (%)	0.45 ± 0.09	0.52 ± 0.08	<0.001	0.882
*f*·*D*^∗^	39.24 ± 10.87	42.05 ± 11.03	0.213	0.813
*K* ^trans^ (min-1)	0.53 ± 0.29	0.92 ± 0.51	<0.001	0.914
*K*_ep_ (min-1)	0.64 ± 0.22	0.78 ± 0.19	0.002	0.894
*V*_*e*_	0.10 (0.05, 0.33)	0.15 (0.08, 0.28)	0.204	0.826
*V*_*p*_	0.08 (0.04, 0.20)	0.10 (0.06, 0.21)	0.351	0.863

**Table 2:** Diagnostic performance of perfusion-related IVIM and DCE parameters to discriminate poor differentiation tumor.

Parameters	AUC	*P* value	95% CI	Sensitivity (%)	Specificity (%)	Cutoff value
*f*	0.728	<0.0001	0.629, 0.813	92.7	43.9	>0.43
*K* ^trans^	0.775	<0.0001	0.680, 0.854	85.4	63.2	>0.53
*K*_ep_	0.710	0.0001	0.609, 0.797	92.7	49.1	>0.60

**Table 3:** Correlations between DCE and IVIM parameters and pathological differentiation grade.

Parameters	Differentiation grade	
	*R*_*s*_	*P* value
*f*	0.289	<0.001
*K* ^trans^	0.471	<0.001
*K*_ep_	0.358	<0.001

## Data Availability

The data used to support the findings of this study are available from the corresponding author upon request.
